The article "Two Pore Channel 2 (TPC2) Inhibits Autophagosomal-Lysosomal Fusion by Alkalinizing Lysosomal pH" was retracted in 2017. Reasons: fabricated or falsified images; manipulated images; ethical violations by an author.

# Two Pore Channel 2 (TPC2) Inhibits Autophagosomal-Lysosomal Fusion by Alkalinizing Lysosomal pH*[Fn FN2]

**DOI:** 10.1074/jbc.M113.484253

**Published:** 2013-07-08

**Authors:** Yingying Lu, Bai-Xia Hao, Richard Graeff, Connie W. M. Wong, Wu-Tian Wu, Jianbo Yue

**Affiliations:** From the ‡ Department of Physiology, University of Hong Kong, Hong Kong, China,; § Department of Anatomy and State Key Laboratory of Brain and Cognitive Sciences, University of Hong Kong, Hong Kong, China, and; ¶ GHM Institute of CNS Regeneration, Jinan University, Guangzhou, China

**Keywords:** Autophagy, Calcium, Calcium Channels, Calcium Intracellular Release, Calcium Signaling, Lysosomes, NAADP, TPC2, pH

## Abstract

Autophagy is an evolutionarily conserved lysosomal degradation pathway, yet the underlying mechanisms remain poorly understood. Nicotinic acid adenine dinucleotide phosphate (NAADP), one of the most potent Ca^2+^ mobilizing messengers, elicits Ca^2+^ release from lysosomes via the two pore channel 2 (TPC2) in many cell types. Here we found that overexpression of TPC2 in HeLa or mouse embryonic stem cells inhibited autophagosomal-lysosomal fusion, thereby resulting in the accumulation of autophagosomes. Treatment of TPC2 expressing cells with a cell permeant-NAADP agonist, NAADP-AM, further induced autophagosome accumulation. On the other hand, TPC2 knockdown or treatment of cells with Ned-19, a NAADP antagonist, markedly decreased the accumulation of autophagosomes. TPC2-induced accumulation of autophagosomes was also markedly blocked by ATG5 knockdown. Interestingly, inhibiting mTOR activity failed to increase TPC2-induced autophagosome accumulation. Instead, we found that overexpression of TPC2 alkalinized lysosomal pH, and lysosomal re-acidification abolished TPC2-induced autophagosome accumulation. In addition, TPC2 overexpression had no effect on general endosomal-lysosomal degradation but prevented the recruitment of Rab-7 to autophagosomes. Taken together, our data demonstrate that TPC2/NAADP/Ca^2+^ signaling alkalinizes lysosomal pH to specifically inhibit the later stage of basal autophagy progression.

## Teaser

**Background:** The role and mechanism of NAADP, an endogenous Ca^2+^ mobilizing nucleotide, in autophagic regulation remain to be determined.

**Results:** Activation of NAADP/TPC2 signaling induced the accumulation of autophagosomes.

**Conclusion:** The NAADP/TPC2 signaling inhibits autophagosomal-lysosomal fusion by alkalinizing lysosomal pH.

**Significance:** Development of agonists or antagonists of NAADP should provide a novel approach to specifically manipulate autophagy.

## Introduction

Macroautophagy (hereafter referred as autophagy) is an evolutionarily conserved catabolic degradation cellular process. Autophagy starts with sequestering of cytoplasmic material, such as misfolded proteins and/or damaged organelles, inside the phagophore followed by the elongation and closure of the autophagosome, a double-membrane vesicle. The matured autophagosome then fuses with the lysosome to create an autolysosome inside which the autophagosome inner membrane and its luminal contents are degraded by lysosomal enzymes for subsequent recycling of macromolecules. Autophagy can also be markedly induced by a wide variety of stresses, such as nutrient starvation, infection, and aging, for cell survival. Dysfunctional autophagy has been associated with wide-ranging human diseases, *e.g.* cancer, neurodegenerative diseases, heart disease, diabetes, and infections (1).

The article "Two Pore Channel 2 (TPC2) Inhibits Autophagosomal-Lysosomal Fusion by Alkalinizing Lysosomal pH" was retracted in 2017. Reasons: fabricated or falsified images; manipulated images; ethical violations by an author.

Autophagy induction is controlled by the ULK1 and ULK2 complexes, and autophagosome formation requires class III phosphatidylinositol 3 kinase (PI3K) complexes. The key autophagy regulator is mTOR Ser/Thr kinase, which negatively regulates autophagy by inhibiting the ULK1/2 complex. Starvation, on the other hand, activates the AMP-activated protein kinase (AMPK) to inactivate mTOR, thereby inducing autophagy. Another key step for autophagy induction is the activation of mammalian Vps34, a class III PI3K. Vps34 is activated by forming a multiprotein complex with beclin-1, UVRAG, and Vps15, to generate phosphatidylinositol 3-phosphate. Two ubiquitin-like conjugation systems, the LC3-II and Atg12-Atg5-Atg16L complex, are essential for the autophagosomal elongation process. The covalent conjugation of Atg12 to Atg5 is catalyzed by the E1-like enzyme Atg7 and the E2-like enzyme Atg10. The conjugation of phosphatidylethanolamine to LC3 is sequentially controlled by the protease Atg4, Atg7, and the E2-like enzyme Atg3. Lipidation of LC3 converts the cytosolic LC3 (LC3-I) to the autophagic vesicle-associated form (LC3-II). Notably, LC3-II is commonly used as a marker of autophagy because lipidated LC3-II exhibits a punctate staining pattern and has faster electrophoretic mobility compared with diffused LC3-I (1, 2). Besides mTOR, other signaling pathways, *e.g.* JNK, Ras, and Ca^2+^, can modulate autophagy as well (3, 4).

Even after extensive research, the regulation and mechanisms of autophagy induction, autophagosome formation and maturation, and especially autophagosomal-lysosomal fusion, remain elusive in mammalian cells. Although autophagosomal-lysosomal fusion is poorly understood, many factors and proteins, including lysosomal pH (5), Rab7 (6), SNAREs (7), the HOPS complex (8), TECPR1 (9), histone deacetylase-6 (10), ubiquilins (11), Hrs (12), OATL1 (13), COP9 signalosome (14), presenilin 1 (15), the ESCRT III complex (16), LAMP1/2 (17), UVRAG (18), p97VCP (19), LRRK2 (20), and HSP70 (21) have been implicated in regulating this process. We have been studying the effects of lysosomal specific ion channels on autophagosomal-lysosomal fusion.

The article "Two Pore Channel 2 (TPC2) Inhibits Autophagosomal-Lysosomal Fusion by Alkalinizing Lysosomal pH" was retracted in 2017. Reasons: fabricated or falsified images; manipulated images; ethical violations by an author.

In vertebrates, three TPC^2^ genes, TPC1, -2, and -3, have been cloned. TPCs contain two putative pore-forming repeats, with each of the repeats containing six transmembrane domains and an intervening pore-forming loop. The transmembrane domain of TPCs is similar to that of voltage-gated Ca^2+^/Na^+^ channels. Interestingly, human and rodent only encode TPC1 and TPC2. TPC2 predominantly localizes on lysosomes, whereas TPC1 is mainly on late endosomes, and TPC3 is thought to be in the recycling endosomes. Ever since their identification, TPCs have become the prime candidates for NAADP-mediated Ca^2+^ release from lysosome-related stores (22–24). NAADP is a metabolite of nicotinamide adenine dinucleotide phosphate (NADP) and is formed by a base-exchange reaction catalyzed by ADP-ribosyl cyclases, which replaces the nicotinamide moiety of NADP with nicotinic acid. NAADP mobilizes Ca^2+^ from acidic lysosome-related stores in a wide variety of cells, from plant to animal, including human (25). Ample evidence indicates that TPC2 forms NAADP-sensitive Ca^2+^-permeable channels in many cell types. TPC2 overexpression promotes NAADP-induced Ca^2+^ release from lysosome-related stores, whereas ablating or knocking-down TPC2 expression blocks NAADP-induced Ca^2+^ release. Moreover, TPC2 knock-out abolishes NAADP-mediated smooth muscle contraction, a well established function of NAADP (26–33). Besides TPC2, other NAADP receptor candidates have been reported in different cell types, including TPC1 in SKBR3 human breast carcinoma (34, 35), TRP mucolipin 1(TRPML1) in coronary arterial myocytes (36, 37), and TRPM2 or ryanodine receptors in T lymphocytes (38, 39). Interestingly, several recent papers found that NAADP does not directly bind to TPC2, suggesting that NAADP first binds to accessory proteins, which subsequently activate TPC2 or other ion channels for Ca^2+^ mobilization depending upon the cell type (40–42).

Previously, two groups found that activation of NAADP/TPC2 signaling increased LC3-II levels (43, 44), and another report found that down-regulation of TPC2 by presenilin decreased LC3-II (45), thus concluding that TPC2 signaling mainly induces the initiation of autophagy. However, here we found that the increased LC3-II levels by TPC2 signaling are not due to the enhanced autophagy activity but result from the inhibition of basal autophagy progression, which leads to the accumulation of autophagosomes. Inhibition of TPC2 signaling either by TPC2 knockdown or by treatment with a NAADP antagonist, on the other hand, facilitates autophagosomal-lysosomal fusion, thereby decreasing LC3-II levels.

The article "Two Pore Channel 2 (TPC2) Inhibits Autophagosomal-Lysosomal Fusion by Alkalinizing Lysosomal pH" was retracted in 2017. Reasons: fabricated or falsified images; manipulated images; ethical violations by an author.

## EXPERIMENTAL PROCEDURES

### 

#### 

##### Antibodies and Reagents

LC3 antibody (antibody from MBL was used in study in the embryonic stem (ES) cells, and the one from Novus was used in the study in HeLa cells; 1:500 for the immunofluorescence analysis and 1:1000 for the Western blotting analysis (WB)), p62 antibody (Novus; 1:1000 WB), cathepsin-L antibody (BD Bioscience; 1:250 WB), Lamp-1 and EGFR antibodies (Santa Cruz; 1:250 WB), Lamp-1 antibody (Cell Signaling; 1:500 immunofluorescence analysis), phospho-mTOR and mTOR antibodies (Cell Signaling; 1:500 WB), GAPDH antibody (Sigma; 1:5000 WB), and TPC2 antibody (a custom rabbit polyclonal antibody against rat TPC2; 1:500 immunofluorescence analysis and 1:1000 WB). Bafilomycin A1, rapamycin, and BAPTA-acetoxymethyl (AM) were all purchased from Sigma. NH_4_Cl was purchased from Merck. Fura-2 AM, dye-quenched (DQ)-BSA-green, lysosensor Green DND-189, and LysoSensor Yellow/Blue DND-160 were purchased from Invitrogen.

##### Cell Culture

HeLa cells (ATCC) were maintained in DMEM (Invitrogen) plus 10% fetal bovine serum (Invitrogen) and 100 units/ml penicillin/streptomycin (Invitrogen) at 5% CO_2_ and 37 °C. ES cells, D3 from Prof. S. Y. Tsang (Chinese University of Hong Kong), and 46C Sox1-GFP from Prof. Austin Smith (University of Cambridge), were normally maintained with feeders (mouse embryonic fibroblasts) in Dulbecco's modified Eagle's medium plus 15% FBS (ES qualified, Invitrogen), 1% nonessential amino acids, 1% penicillin-streptomycin, 0.2% 2-mercaptoethanol, 1000 units/ml leukemia inhibitory factor. Cells are passaged every 2 days. Before any experimental procedures, ES cells are cultured in feeder-free ES medium containing leukemia inhibitory factor on gelatin-coated plates for two passages. The pluripotency of ES cells are periodically assessed by alkaline phosphatase assay and Oct4 immunostaining.

##### TPC2 shRNA, TPC2, GFP-LC3, RFP-GFP-LC3 Lentivirus Production and Infection

Three optimal 21-mers were selected in the mouse TPC2 genes (supplemental Table S1). One 21-mer was selected in the GFP gene as a control. These sequences were then cloned into the pLKO.1 vector for expressing shRNA. Likewise, a rat TPC2, GFP-LC3, or RFP-GFP-LC3 (tfLC3) cDNA was cloned into pLenti-CMV-Puro-DEST (Addgene). The shRNA, TPC2, GFP-LC3, or tfLC3 lentivirus production was performed in 293T cells. For infection, cells were plated at a density of 3 × 10^5^ cells/well in 6-well plates. On the next day, 100-μl pools of shRNAs lentivirus were added to the cells in fresh medium containing 8 μg/ml Polybrene. Two days later cells infected with shRNA lentiviruses were selected in fresh medium containing puromycin (3 μg/ml) for 3–5 days. The puromycin-resistant cells were pooled, and the knockdown efficiency was verified by both quantitative real-time RT-PCR and/or Western blot analyses.

The article "Two Pore Channel 2 (TPC2) Inhibits Autophagosomal-Lysosomal Fusion by Alkalinizing Lysosomal pH" was retracted in 2017. Reasons: fabricated or falsified images; manipulated images; ethical violations by an author.

##### Intracellular Ca^2+^ Measurement

Intracellular Ca^2+^ in HeLa cells were measured as described previously (46, 47). Briefly, cells were cultured in 24-well plates at the density of 5 × 10^4^ cells/well in regular DMEM medium overnight. Before Ca^2+^ measurement, cells were incubated for 30 min in Hanks' balanced salt solution containing 4 μm Fura-2 AM and 0.04% F127 in the dark at room temperature. The cells were then washed with Hanks' balanced salt solution three times and incubated at room temperature for another 10 min. Cells were put on the stage of an Olympus epifluorescence microscope and visualized using a 20× objective. Fluorescence images were obtained by alternate excitation at 340 and 380 nm with emission set at 510 nm. Images were collected by a CCD camera every 3 s. Finally, the images were saved and analyzed by Cell R imaging software.

##### Western Blot Analysis

Western blot analysis was performed as described previously (48, 49). Briefly, cells were lysed in an ice-cold EBC lysis buffer (50 mm HEPES at pH 7.5, 0.15 m NaCl, 1 mm EDTA, 1% Nonidet P-40, 150 μm PMSF, 10 mm NaF, 10 ng/ml leupeptin, 1 mm DTT, and 1 mm sodium vanadate) and passed through a 21-gauge needle several times to disperse any large aggregates. Protein concentrations of the cell lysates were determined by Bradford protein assay. 30–100 μg of protein per lane was diluted in the standard SDS sample buffer and subjected to electrophoresis on SDS-PAGE gels. Proteins were then transferred to an Immobilon PVDF membrane (Millipore, Billerica, MA*),* blocked with 5% milk in TBST (20 mm Tris, 150 mm NaCl, pH 7.6), and incubated with the primary antibody overnight. After washing with TBST, the blots were probed with a secondary antibody (1:5000 dilution) for detection by chemiluminescence.

##### RNA Isolation and Quantitative Real-time RT-PCR

Total RNA was extracted from HeLa cells or mouse ES cells at various stages of neural differentiation using an RNA extraction kit (Invitrogen). The quantitative real-time RT-PCR using the SuperScript® III Platinum® One-Step Q-RT PCR Kit (Invitrogen) was performed in a MiniOpticon^TM^ Real-time PCR Detection System (Bio-Rad) according to the manufacturer's instructions. The primers for detecting tpc2 and GAPDH mRNAs are listed in supplemental Table S1. Relative gene expression was normalized to GAPDH expression.

The article "Two Pore Channel 2 (TPC2) Inhibits Autophagosomal-Lysosomal Fusion by Alkalinizing Lysosomal pH" was retracted in 2017. Reasons: fabricated or falsified images; manipulated images; ethical violations by an author.

##### Immunofluorescence Staining Analysis

Immunofluorescence staining analysis was performed as described previously (50). Briefly, infected or transfected cells grown on coverslips were fixed for 20 min with 4% paraformaldehyde at room temperature and washed twice with PBS, and nuclei were labeled with DAPI to identify each individual cell. For immunostaining analysis, fixed cells were further blocked with 1% goat serum, 1% BSA, 0.1% Triton X-100 in PBS for 1 h. Thereafter, the cover glasses were incubated with primary antibodies for 2 h, washed, and incubated with a secondary antibody (Alexa Fluor® 488 or 568 goat anti-mouse or rabbit IgG, Invitrogen; 1:1000 dilution) for 1 h. Images were captured under a Zeiss LSM710 confocal microscope with a Plan-Apochromat ×63/1.40 oil differential interference contrast objective. Images were processed and analyzed with Zeiss ZEN software.

##### Transmission Electron Microscopy

Cell preparation for transmission electron microscopy was performed as described previously (51). Briefly, cells were washed in PBS and fixed in 2% formaldehyde and 2.5% glutaraldehyde for 2 h. After fixation, cells were pelleted, transferred to glass slides, and allowed to dry on a hotplate at 37 °C before embedding in 2% agarose solution. Agarose-embedded blocks were then fixed in the same fixative solution at 4 °C for 4 h. Thereafter, the blocks were washed three times with PBS and post-fixed with 1% osmium tetroxide solution in PBS at 4 °C overnight. Blocks were subsequently dehydrated in graded ethanol, embedded in pure Epon, and kept at 60 °C for 3 days. Ultrathin sections (∼90 nm) were cut and stained with 8% uranyl acetate and lead citrate before observation under electron microscope.

For immunoelectron microscopy, cells were incubated with primary antibody (rabbit anti-LC3 antibody, 1:100) at 4 °C overnight. After incubation in the primary antibody, the cells were incubated in biotinylated secondary antibody (biotinylated goat anti-rabbit IgG antibody, 1:200) for 40 min at room temperature. Cells were then incubated in ABC reagents (Vectastain ABC kit) for 60 min at room temperature, sequentially, followed by incubating in 0.05% diaminobenzidine and 0.03% H_2_O_2_ for 3–5 min until a brown reaction product was observed. The stained cells were then processed to transmission electron microscopy study as described above.

##### Neural Differentiation

The *in vitro* neural differentiation of mouse ES cells was performed as described previously (52). Briefly, feeder-free ES cells were plated onto 0.1% gelatin-coated plates at a density of 0.8∼1 × 10^4^ cells/cm^2^ in N2B27 medium (1:1 mixture of DMEM/F12 and neurobasal medium supplemented with N2 and B27 plus 50 μg/ml bovine serum albumin (BSA) fraction V and 20 μm β-mercaptoethanol). The medium was changed every other day until day 8.

The article "Two Pore Channel 2 (TPC2) Inhibits Autophagosomal-Lysosomal Fusion by Alkalinizing Lysosomal pH" was retracted in 2017. Reasons: fabricated or falsified images; manipulated images; ethical violations by an author.

##### Lysosomal pH Measurement

LysoSensor Green DND-189 is commonly used to qualitatively measure the pH of acidic organelles, such as lysosomes, which become more fluorescent in acidic environments and less fluorescent in alkaline environments (53). Briefly, cells were loaded with 1 μm LysoSensor Green DND-189 in prewarmed regular medium for 20 min at 37 °C. Then the cells were washed twice with PBS and immediately analyzed by flow cytometry (collecting FL1 fluorescence, and 10,000 cells were collected for each sample) or in a microplate reader (excitation/emission = 485/530 nm) in triplicate.

Quantification of lysosomal pH was performed using a ratiometric lysosomal pH dye LysoSensor Yellow/Blue DND-160. The pH calibration curve was generated as described previously (54). Briefly, cells were trypsinized and labeled with 2 μm LysoSensor Yellow/Blue DND-160 for 30 min at 37 °C in regular medium, and excessive dye was washed out using PBS. The labeled cells were treated for 10 min with 10 μm monensin and 10 μm nigericin in 25 mm MES calibration buffer, pH 3.5–6.0, containing 5 mm NaCl, 115 mm KCl, and 1.2 mm MgSO_4_. Quantitative comparisons were performed in a 96-well plate, and the fluorescence was measured with a microplate reader at 37 °C. Light emitted at 440 and 535 nm in response to excitation at 340 and 380 nm was measured, respectively. The ratio of light emitted with 340- and 380-nm excitation was plotted against the pH values in MES buffer, and the pH calibration curve for the fluorescence probe was generated from the plot using Microsoft Excel.

##### NH_4_Cl Chase Assay

HeLa cells were seeded in regular DMEM medium overnight and then incubated with 100 μm NH_4_Cl in regular DMEM medium without sodium bicarbonate for 20 min at 37 °C. Thereafter, NH_4_Cl was removed, and the cells were washed with regular medium without sodium bicarbonate continuously and thoroughly. Samples were collected at the indicated time and finally analyzed by Western blotting analyses or for pH measurement in a microplate reader.

##### Statistical Analysis

All data were presented as the means ± S.E. Student's *t* test was performed to determine the differences among grouped data. * denotes statistically significant with *p* < 0.05.

## RESULTS

### 

#### 

##### Reconstitution of NAADP Competence in HeLa Cells by TPC2 Overexpression

HeLa cell line is an autophagy-competent cell line (supplemental Fig. S1, *A* and *B*). Yet HeLa cells are not responsive to NAADP-induced Ca^2+^ changes (Fig. 1*A*), which might be due to the low expression level of endogenous TPC2 (supplemental Fig. S1*C*). We thus first constructed a stable rat TPC2-overexpressing HeLa cell line by lentiviral infection. As shown in Fig. 1*B*, TPC2 was overexpressed in the lysosome as indicated by its co-localization with the lysosomal marker Lamp1 in a subset of cellular puncta (the TPC2-positive vesicles were actually enlarged in some cells as compared with the control). Likewise, the HeLa cells expressing a rat TPC2 249L/P mutant, in which a highly conserved leucine residue within a putative pore region of rat TPC2 was mutated to proline (34), were constructed by lentiviral infection (Fig. 1*B*). A cell permeant NAADP analog, NAADP-AM (55), induced Ca^2+^ release only in wild type TPC2-overexpressing HeLa cells and not in TPC2 249L/P mutant-expressing cells (Fig. 1*A*) and displayed a characteristic bell-shaped dose-response curve due to the activation of its receptor by low concentrations of NAADP and its desensitization by high concentrations of NAADP. The induced Ca^2+^ release was markedly inhibited by preincubation with Ned-19 (56), an NAADP antagonist (Fig. 1*C*). These data indicated that HeLa cells can be reconstituted to be NAADP competent via TPC2 overexpression.

The article "Two Pore Channel 2 (TPC2) Inhibits Autophagosomal-Lysosomal Fusion by Alkalinizing Lysosomal pH" was retracted in 2017. Reasons: fabricated or falsified images; manipulated images; ethical violations by an author.

**FIGURE 1.** **Reconstitution of NAADP-competent HeLa cells by overexpressing TPC2.** *A*, NAADP-AM (100 nm) only induced Ca^2+^ release in wild type, but not in an inactive mutant, TPC2-overexpressing HeLa cells. *B*, shown is localization of Lamp1-RFP, TPC2, and TPC2 249L/G in HeLa cells. A rabbit polyclonal TPC2 antibody was used to detect overexpressing TPC2. *Scale bar* = 5 μm. *C*, NAADP-AM induced Ca^2+^ release in TPC2-overexpressing HeLa cells, which was markedly inhibited by Ned-19 (10 μm). Note the bell-shaped concentration dependence curve for NAADP-AM. Quantification of the [Ca^2+^]*_i_* peak induced by drug treatment in *A* and *C* is expressed as the mean ± S.E., *n* = 30–40 cells. The *asterisk* indicates the results of *t* test analysis; *p* < 0.05.

##### Inhibition of Autophagic Flux by TPC2 in HeLa Cells

Strikingly, under the electron microscope, large numbers of autophagic vacuoles were observed in TPC2-overexpressing HeLa cells maintained in normal (nutrient-rich) culture conditions but not in control cells (Fig. 2*A*). Similar to previous reports (43), lipidated LC3-II, a reliable autophagosome marker, was markedly increased in TPC2-overexpressing cells compared with that in TPC2 mutant expressing or control HeLa cells (Fig. 2*B*). Interestingly, p62, an autophagic substrate (57), was also accumulated in TPC2-overexpressing cells compared with that in control HeLa cells, suggesting that TPC2 overexpression results in a defect of autophagic degradation instead of simply promoting autophagy (Fig. 2*B*). Consistently, endogenous LC3-II puncta (Fig. 2*C*) or GFP-LC3 puncta (Fig. 2*D* and supplemental Fig. S1*A*) were greatly increased in TPC2-overexpressing cells and did not co-localize with Lamp1, which was similar to the cells treated with bafilomycin (BAF), an inhibitor of the vacuolar proton pump that blocks the fusion of autophagosomes with lysosomes (58). These data suggest that these LC3-II puncta present in TPC2-overexpressing cells are autophagosomes, not autolysosomes.

The article "Two Pore Channel 2 (TPC2) Inhibits Autophagosomal-Lysosomal Fusion by Alkalinizing Lysosomal pH" was retracted in 2017. Reasons: fabricated or falsified images; manipulated images; ethical violations by an author.

**FIGURE 2.** **TPC2 overexpression induced a defect in autophagic degradation in HeLa cells.** *A*, large numbers of autophagic vacuoles were observed in TPC2-overexpressing cells, but not in control cells, under electron microscope. *B*, wild type, not an inactive mutant, TPC2 overexpression induced the accumulation of both LC3-II and p62. *C*, wild type, not an inactive mutant, TPC2 overexpression markedly induced endogenous LC3-II puncta (*green*) in HeLa cells, which were not colocalized with RFP-Lamp1. *Scale bar* = 5 μm. Quantification of LC3 puncta is expressed as the mean ± S.E., *n* = ∼80 cells. The *asterisks* indicate the results of *t* test analysis; *p* < 0.05. *D*, starvation induced LC3 puncta, some of which were colocalized with LAMP1 puncta, whereas the LC3 puncta induced by bafilomycin or TPC2 expression failed to co-localize with LAMP1 in RFP-LAMP1/GFP-LC3 HeLa cells. *Scale bar* = 10 μm.

Because it is possible that the accumulation of LC3-II in TPC2-overexpressing cells is partly due to the increased early autophagic activity, we briefly (1 h) treated control or TPC2-overexpressing HeLa cells with BAF in normal or serum-free medium. We reasoned that BAF treatment could further induce the accumulation of LC3-II and p62 if TPC2, like starvation, promotes early autophagic progression. However, BAF treatment (1 h) only induced the accumulation of LC3-II and p62 in control cells, not in TPC2-overexpressing cells, regardless of whether cells were in normal or starvation states (Fig. 3*A* and supplemental Fig. S1*B*). This suggests that TPC2 is not involved in early autophagy induction. Also notably, starvation not only induced the accumulation of LC3-II but also decreased p62 in both control and TPC2-overexpressing cells (comparing *lanes 5* and *6* in Fig. 3*A*), suggesting that TPC2 overexpression only inhibits but does not abolish the fusion of autophagosomes with lysosomes.

**FIGURE 3.** **TPC2 overexpression did not affect the early autophagic progression in HeLa cells.** *A*, bafilomycin (10 nm, 1 h) only induced the accumulation of LC3-II and p62 in control, not TPC2-overexpressing, HeLa cells, whereas starvation induced autophagic progression in both cells. The quantification of the *four boxed lanes* is shown. *B*, starvation (60 min) induced RFP-ATG5 puncta, most of which were not colocalized with GFP-LC3 puncta, in both control and TPC2-overexpressing HeLa cells. *C*, TPC2 failed to induce LC3-II and p62 in ATG5 knockdown cells. *D*, ATG5 knockdown markedly inhibited TPC2-induced accumulation of LC3-II and p62 in HeLa cells. *E*, TPC2 overexpression did not affect p62 incorporation into autophagosome in HeLa cells. *Scale bar* = 10 μm.

The article "Two Pore Channel 2 (TPC2) Inhibits Autophagosomal-Lysosomal Fusion by Alkalinizing Lysosomal pH" was retracted in 2017. Reasons: fabricated or falsified images; manipulated images; ethical violations by an author.

After the initiation of the phagophores, autophagosomes undergo a stepwise maturation process from early to late autophagosomes, which ultimately fuse with lysosomes to form autolysosomes. Any missteps during the maturation process could lead to the accumulation of autophagosomes (1). Therefore, we next assessed whether TPC2 signaling compromises early autophagosome formation. To do so, GFP-LC3 or GFP-LC3/TPC2-expressing HeLa cells were transfected with RFP-ATG5. Under normal conditions (nutrient-rich), ATG5 was diffuse throughout the cytoplasm in both control and TPC2-overexpressing HeLa cells, again suggesting that TPC2 does not induce autophagy. Starvation (60 min), on the other hand, markedly induced puncta formation of ATG5, some of which were not colocalized with LC3 in both cell types (Fig. 3*B*). These data suggest that TPC2 signaling does not inhibit the early autophagosome(s) maturation.

Subsequently, we tested whether the accumulated autophagosomes in TPC2-overexpressing HeLa cells are the result of basal cellular autophagy activity. To do so, we knocked-down ATG5, which is required for the elongation and closure of autophagosomes in both control and TPC2-overexpressing HeLa cells (supplemental Fig. S2*A*). As expected, not only did TPC2 overexpression in ATG5-knockdown cells fail to induce autophagosome(s) accumulation (Fig. 3*C* and supplemental Fig. S2*B*), but also knockdown of ATG5 in TPC2-overexpressing cells markedly decreased the accumulated LC3-II and p62 (Fig. 3*D*). These results place TPC2 downstream of ATG5 in autophagy regulation and again suggest that TPC2 overexpression does not completely block the fusion of autophagosomes with lysosomes.

p62, as a cargo receptor for some ubiquitinated proteins, is first incorporated into autophagosomes before being targeted to lysosomes for degradation (59). Therefore, it is also necessary to clarify whether accumulated p62 in TPC2-overexpressing cells is due to the defects in cargo incorporation into autophagosomes. As shown in Fig. 3*E*, under normal culture conditions, p62 puncta were already markedly accumulated in TPC2-overexpressing cells compared with control cells, and most of them were co-localized with LC3-II. Moreover, similar to control cells, starvation further induced LC3-II puncta and p62 puncta in TPC2-overexpressing cells (Fig. 3*E*). This indicates that TPC2 does not prevent p62 incorporation into autophagosomes and suggests that accumulated p62 in TPC2-overexpressing cells is due to the defects in later stages of autophagy.

The article "Two Pore Channel 2 (TPC2) Inhibits Autophagosomal-Lysosomal Fusion by Alkalinizing Lysosomal pH" was retracted in 2017. Reasons: fabricated or falsified images; manipulated images; ethical violations by an author.

##### Inhibition of the Fusion between Autophagosomes and Autolysosomes by NAADP/TPC2 Signaling in HeLa Cells

To further differentiate autophagosomes and autolysosomes during autophagy, we infected the control or TPC2-overexpressing HeLa cells with lentiviruses carrying expression cassettes that encode RFP-GFP-LC3 (tfLC3), in which RFP and GFP are tandem-tagged to the N terminus of LC3 (60). Before fusion with lysosomes, the LC3-II-positive autophagosomes are shown by both GFP and RFP signals as yellow puncta, and after fusion, autolysosomes are shown by only RFP signals as red only puncta because GFP loses its fluorescence in acidic pH. As expected, yellow puncta (autophagosomes) were markedly increased with few red puncta signals (autolysosomes) in wild type, not mutant, TPC2-overexpressing cells, which was similar to the effects of BAF in control cells. In contrast, starvation dramatically increased both yellow and red puncta in control cells (Fig. 4, *A* and *B*). We further performed immunoelectron microscopy analyses to distinguish autophagosomes from autolysosomes in control and TPC2-overexpressing HeLa cells (Fig. 4*C*). The cells were incubated with anti-LC3 antibody followed by diaminobenzidine staining and were subsequently subjected to EM analyses. Two types of autophagic structures were quantified: autophagosomes whose surfaces are LC3-positive (Fig. 4*C1*) and autolysosomes whose inside are LC3-positive (Fig. 4*C2*). Consistently, the numbers of autophagosomes in TPC2-overexpressing cells were significantly more than those in control cells, whereas autolysosomes were hard to find in both control and TPC2-overexpressing cells (the *bottom panel* of Fig. 4*C*). Thus, these data clearly demonstrate that TPC2 overexpression inhibits the fusion between autophagosomes and autolysosomes, thereby resulting in a marked accumulation of autophagosomes.

**FIGURE 4.** **TPC2 signaling inhibited the progression of autophagy in HeLa cells.** *A*, HeLa cells were transfected with a RFP-GFP tandem fluorescent-tagged LC3 (tfLC3) plasmid. TPC2 overexpression induced *yellow* puncta with few *red*-only puncta signals in cells. In contrast, starvation dramatically increased both yellow and red puncta in control cells. *Scale bar* = 10 μm. *B*, quantitation of % of yellow puncta or red only puncta/per cell of *A* are expressed as the mean ± S.E., *n* = ∼ 80 cells. The *asterisks* indicate the results of *t* test analysis; *p* < 0.05. *C*, control and TPC2-overexpressing cells were processed for immunoelectron microscopy analyses. *C1*, shown are representative autophagosomal structures, whose surfaces are LC3-positive, in TPC2-overexpressing HeLa cells; *C2*, shown are representative autolysosomal structures, whose inside are LC3-positive, in TPC2-overexpressing HeLa cells. Quantitation of autophagosomes and autolysosomes per cell are expressed as the mean ± S.E., *n* = ∼ 40 cells (*bottom panel*). *ns*, not significant. *D*, NAADP-AM (100 nm) increased the accumulation of both LC3-II and p62 only in TPC2-overexpressing, not the control, HeLa cells. *E*, Ned-19 (10 μm) decreased the levels of both LC3-II and p62 in TPC2-overexpressing, but not the control, HeLa cells.

The article "Two Pore Channel 2 (TPC2) Inhibits Autophagosomal-Lysosomal Fusion by Alkalinizing Lysosomal pH" was retracted in 2017. Reasons: fabricated or falsified images; manipulated images; ethical violations by an author.

Because TPC2 is a NAADP-sensitive Ca^2+^-permeable channel in lysosomes, we examined the effects of NAADP-AM on the fate of autophagosomes in TPC2-overexpressing cells. As shown in Fig. 4*D* and supplemental Fig. S3*A*, NAADP-AM indeed further induced the accumulation of both LC3-II and p62 only in TPC2-overexpressing HeLa cells. On the other hand, treatment with Ned-19, a NAADP antagonist, decreased the levels of both LC3-II and p62 only in TPC2-overexpressing cells (Fig. 4*E*, supplemental Fig. S3, *B* and *C*). Moreover, Ned-19 increased the red LC3 puncta (autolysosomes), whereas it decreased the yellow LC3 puncta (autophagosomes) in TPC2/RFP-GFP-LC3 co-expressing HeLa cells (Fig. 4, *A* and *B*). Taken together, our results further demonstrate that the activation of NAADP/TPC2 signaling compromises autophagy progression, resulting in autophagosome accumulation.

##### Inhibition of Autophagic Flux by Endogenous TPC2 Signaling in Mouse Embryonic Stem Cells

Upon withdrawal of self-renewal stimuli, mouse ES cells can spontaneously and robustly differentiate into neural progenitors in adherent monoculture (61). Interestingly, autophagy was markedly induced during neural differentiation of mouse ES cells (Fig. 5*A* and supplemental Fig. S4*A*). TPC2 is detectable in mouse ES cells (Fig. 5*B*), and quantitative RT-PCR analyses showed that the expression of TPC2 mRNA was dynamically regulated during neural differentiation of mouse ES cells (supplemental Fig. S4*B*). Thus, we used lentivirus-mediated short hairpin RNA (shRNA) or cDNA to stably knockdown the expression of TPC2 (Fig. 5*B*) or to overexpress TPC2 (Fig. 5*C*), respectively, in mouse ES cells.

The article "Two Pore Channel 2 (TPC2) Inhibits Autophagosomal-Lysosomal Fusion by Alkalinizing Lysosomal pH" was retracted in 2017. Reasons: fabricated or falsified images; manipulated images; ethical violations by an author.

**FIGURE 5.** **TPC2 signaling inhibited the progression of autophagy during neural differentiation of mouse ES cells.** *A*, *in vitro* neural differentiation of mouse ES cells initiated by monolayer adherent culture markedly induced LC3-II in D3 mouse ES cells. *B*, TPC2 knockdown by shRNA in ES cells was determined by TPC2 immunoblot analyses. *C*, TPC2 is expressed in lysosome-related organelles, as it is co-localized with LysoTracker (*red*). *Scale bar* = 50 μm. *D*, TPC2 overexpression induced accumulation of LC3-II in ES cells during neural differentiation. Treatment with bafilomycin (100 nm) only induced the accumulation of LC3-II in control cells but not in TPC2-overexpressing cells. *E*, TPC2 knockdown decreased the accumulation of LC3-II in ES cells during neural differentiation. Treatment with bafilomycin (100 nm) induced the accumulation of LC3-II in both control and TPC2 knockdown cells. *F*, mouse D3 ES cells were infected with RFP-GFP tandem fluorescent-tagged LC3 (tfLC3) lentiviruses. TPC2 overexpression induced yellow puncta with few red only puncta signals, whereas TPC2 knockdown increased the red-only puncta in ES cells after 4 days of neural differentiation. Quantification of at least 50 cells from three independent experiments is expressed as the mean ± S.E. and shown in the *right columns*. The *asterisks* indicate the results of *t* test analysis; *p* < 0.05. *Scale bar* = 10 μm.

The control scramble-shRNA-infected, TPC2-knockdown, or TPC2-overexpressing cells were then induced to differentiate into neural lineages after the monolayer culture protocol. Similar to HeLa cells, the LC3-II level was markedly accumulated in differentiated TPC2-overexpressing ES cells as compared with that in differentiated control ES cells, and BAF treatment only increased LC3-II levels in control but not in TPC2-overexpressing ES cells (Fig. 5*D* and supplemental Fig. S4*H*). On the other hand, LC3-II levels (Fig. 5*E*, supplemental Fig. S4, *C* and *F*) or LC3 puncta (supplemental Fig. S4, *D* and *E*) were significantly decreased in differentiated TPC2 knockdown ES cells compared with those in control ES cells. Two opposite mechanisms can lead to less LC3-II level or LC3 puncta in TPC2 knockdown cells; a decrease in autophagic induction causes less LC3-II lipidation, or an enhanced fusion between autophagosome and lysosome leads to a faster LC3-II degradation. Interestingly, BAF treatment further increased LC3-II in TPC2 knockdown cells to a level similar to that in control cells (Fig. 5*E* and supplemental Fig. S4*G*), suggesting that the decreased LC3-II level in TPC2 knockdown cells during differentiation is not due to inhibition of autophagic induction but because of the enhanced autophagy progression leads to faster LC3-II degradation. To further assess the possibility that TPC2 knockdown facilitates the fusion between autophagosome and lysosome in order to result in decreased LC3-II levels during differentiation, the tfLC3 was again utilized to distinguish autophagosomes from autolysosomes in differentiated ES cells. Not surprisingly, in tfLC3-expressing ES cells during neural differentiation, more yellow LC3 puncta (autophagosomes) existed in TPC2-overexpressing cells, whereas more red-only LC3 puncta (autolysosomes) appeared in TPC2 knockdown cells (Fig. 5*F*), indicating that autophagosomal-lysosomal fusion is indeed facilitated by TPC2 knockdown but inhibited by TPC2 overexpression. Clearly, these data further demonstrate that the endogenous TPC2 signaling inhibits the fusion between autophagosomes and autolysosomes as well. In addition, we found that TPC2 knockdown facilitated mouse ES cells to differentiate into neural progenitors, whereas TPC2 overexpression inhibited mouse ES cells differentiated into neural progenitors (61).

The article "Two Pore Channel 2 (TPC2) Inhibits Autophagosomal-Lysosomal Fusion by Alkalinizing Lysosomal pH" was retracted in 2017. Reasons: fabricated or falsified images; manipulated images; ethical violations by an author.

##### The Effects of mTOR on TPC2-induced Autophagy Inhibition

The mTOR kinase is one of the key regulators for autophagy, and the activation of mTOR complex 1 occurs at the surface of lysosomes and requires v-ATPase activity (62–64). Moreover, increased mTOR activity is found to be essential for termination of autophagy and reformation of lysosomes (65), and it has recently been shown that ATP activates mTOR to inhibit TPC2 gating (66). We, therefore, assessed whether TPC2 inhibits the fusion between autophagosomes and autolysosomes via mTOR. Unexpectedly, TPC2 overexpression in HeLa cells not only failed to affect mTOR activity but also had no effect on the ability of starvation to inhibit mTOR (Fig. 6*A* and supplemental Fig. S5*B*). Notably, inhibition of mTOR induced by starvation in TPC2-overexpressing cells was accompanied by not only the increase of LC3-II but also the decrease of p62, suggesting that mTOR inhibition does not increase the ability of TPC2 to inhibit autophagy (Fig. 6*A*). Similarly, treatment of cells with rapamycin (50 μm), an mTOR inhibitor, for 3 h increased LC3-II levels and decreased p62 levels in both control and TPC2-overexpressing cells (Fig. 6*B*). Therefore, these data suggest that TPC2 signaling suppresses autophagy maturation independent of mTOR.

**FIGURE 6.** **Ca^2+^, not mTOR, was involved in TPC2-induced autophagosome accumulation in HeLa cells.** *A*, starvation induced LC3-II levels and promoted the degradation of p62 in both control and TPC2-overexpressing HeLa cells accompanied with the inactivation of mTOR. TPC2-induced accumulation of LC3-II and p62 was decreased by Ned-19 (10 μm). *B*, treatment of cells with rapamycin (50 μm) for 3 h promoted autophagy in both control and TPC2-overexpressing cells. *C* and *D*, BAPTA-AM (20 μm) decreased the levels of LC3-II and p62 (*C*) and LC3-II puncta (*D*) in TPC2-overexpressing HeLa cells. Quantification of LC3 puncta is expressed as the mean ± S.E., *n* = ∼ 50 cells. The *asterisk* indicates the results of *t* test analysis; *p* < 0.05. *Scale bar* = 10 μm.

The article "Two Pore Channel 2 (TPC2) Inhibits Autophagosomal-Lysosomal Fusion by Alkalinizing Lysosomal pH" was retracted in 2017. Reasons: fabricated or falsified images; manipulated images; ethical violations by an author.

##### The Effects of Ca^2+^ on TPC2-induced Autophagy Inhibition

NAADP can induce Ca^2+^ release from lysosomes (25), and we found that NAADP treatment actually inhibited autophagosomal-lysosomal fusion (Fig. 4*C* and supplemental Fig. S3*A*). Thus we next examined whether NAADP/TPC2 signaling suppresses autophagy progression via Ca^2+^ release from lysosomes. As shown in Fig. 6*C*, after 1 or 2 h of treatment of cells with BAPTA-AM, a Ca^2+^ chelator, both LC3-II and p62 were markedly decreased in TPC2-overexpressing HeLa cells but not in control cells. Similarly, BAPTA-AM treatment for 1 h significantly decreased LC3-II puncta in TPC2-overexpressing HeLa cells (Fig. 6*D*). Collectively, these data suggest that the inhibition of autophagy progression by NAADP/TPC2 is dependent on Ca^2+^.

##### TPC2 on Lysosomal pH in HeLa and Mouse ES Cells

Interestingly, brief treatment of cells with BAF (∼1 h) failed to further induce the accumulation of LC3-II and p62 in TPC2-overexpressing cells (Fig. 3*A* and supplemental Fig. S5*A*), yet longer treatment with BAF (>3 h) actually further induced the accumulation of these two proteins (supplemental Fig. S5, *A* and *B*). Considering that BAF blocks autophagosomal-lysosomal fusion by raising lysosomal pH via inhibiting the V-proton ATPase and that it has been previously shown that NAADP increases the pH of acidic Ca^2+^ stores in sea urchin egg (67, 68), we speculated that TPC2 overexpression might increase lysosomal pH as well. We first applied LysoSensor Green DND-189 (p*K_a_* = ∼ 5.2) to qualitatively measure lysosomal pH (53). LysoSensor Green DND-189 permeates cell membranes and accumulates in acidic intracellular organelles, and its fluorescence increases or decreases in acidic or alkaline environments, respectively. As shown in Fig. 7*A*, supplemental Fig. S5, *C* and *D*, TPC2 overexpression indeed raised lysosomal pH in HeLa cells, which was similar to that by 1 h of BAF treatment but was less than that by 3 h of BAF treatment. This also explains why only 3 h, not 1 h, of BAF treatment further induced the accumulation of LC3-II and p62 in TPC2-overexpressing HeLa cells (supplemental Fig. S5, *A* and *B*). We further quantified lysosomal pH by dual-emission ratio imaging of LysoSensor Yellow/Blue DND-160-stained cells (supplemental Fig. S5*E*) and found that lysosomal pH in TPC2-overexpressing HeLa cells was increased from pH 4.9 in control cells to pH 5.2 (Fig. 7*B*). Similar results were observed in mouse ES cells (Fig. 7, *C* and *D*). In addition, NAADP-AM transiently raised lysosomal pH only in TPC2-overexpressing HeLa cells (supplemental Fig. S5*F*), which correlated with its effects on LC3-II accumulation (Fig. 3*D*). Next, we assessed whether reacidifying lysosomes in TPC2-overexpressing HeLa cells could relieve the fusion blockage of autophagosomes and lysosomes. An established ammonium chloride (NH_4_Cl) pulse-wash technique was adopted to artificially acidify lysosomal pH (69). To do so, cells were initially incubated with NH_4_Cl. The accumulation of ammonia in lysosomes resulted in an increase of lysosomal pH, which was indicated by a drop of LysoSensor Green DND-189 fluorescence in NH_4_Cl pulsing cells compared with that in cells without NH_4_Cl pulsing (time 0 in Fig. 7*E*). When NH_4_Cl was removed from the medium by thorough washing, the efflux of ammonia caused the pH in the lysosomes to drop rapidly and transiently reach a value lower than that before the ammonium chloride was added, which was indicated by the increases of LysoSensor Green DND-189 fluorescence in NH_4_Cl-pulsed cells after washing (Fig. 7*E*). The transient reacidified lysosomal pH, produced after washing out ammonium chloride, mitigated the fusion blockage in TPC2-overexpressing cells (Fig. 7*F*). Taken together, these data clearly demonstrate that TPC2 signaling suppresses autophagosomal-lysosomal fusion by alkalizing the lysosomal pH.

The article "Two Pore Channel 2 (TPC2) Inhibits Autophagosomal-Lysosomal Fusion by Alkalinizing Lysosomal pH" was retracted in 2017. Reasons: fabricated or falsified images; manipulated images; ethical violations by an author.

**FIGURE 7.** **TPC2 signaling increased lysosomal pH to suppress autophagy progression.** *A*, TPC2 overexpression or BAF treatment induced an increase of lysosomal pH in HeLa cells as determined by FACS analyses of Lysosensor DND-189-stained cells. *B*, quantification of lysosomal pH in control and TPC2-overexpressing HeLa cells as determined by dual-emission ratio imaging of LysoSensor Yellow/Blue DND-160-stained cells. *C* and *D*, TPC2 overexpression or BAF treatment induced an increase of lysosomal pH in D3 ES cells as determined by FACS analyses (*C*) and microplate reader measurement (*D*) of Lysosensor DND-189-stained cells. *E*, washing out NH_4_Cl in both control and TPC2-overexpressing HeLa cells after pulsing with NH_4_Cl (100 μm) for 20 min transiently reacidified lysosomal pH. The data are expressed as the mean ± S.D.; *n* = 4. *F*, washing out NH_4_Cl decreased the accumulation of LC3-II and p62 in TPC2-overexpressing cells after been pulsing with NH_4_Cl (100 μm) for 20 min. The *first lanes* show samples without NH_4_Cl pulsing. The graph in *B* and *D* represents data from three independent experiments, and the data are expressed as the mean ± S.D.; *n* = 3. The *asterisks* indicate the results of *t* test analysis; *p* < 0.05.

##### TPC2 on Rab7 Recruitment to Autophagosomes

Rab7, a small GTPase, is required for autophagosome-lysosome fusion (6). We, thus, assessed the effects of TPC2 overexpression on the localization of Rab7 by transfecting RFP-Rab7 into GFP-LC3 or GFP-LC3/TPC2-overexpressing HeLa cells. We found that starvation induced the co-localization of Rab7 with both GFP-LC3 and Lamp1 in control cells (Fig. 8*A*). On the other hand, RFP-Rab7 puncta were colocalized with Lamp1, but few of them were colocalized with LC3-GFP in TPC2-overexpressing cells (Fig. 8*B*). Next, we assessed whether transient reacidified lysosomal pH by NH_4_Cl pulse-wash in TPC2-overexpressing HeLa cells restores the association of Rab7 with autophagosomes. As shown in Fig. 8*C*, in the majority (⅔) of TPC2-overexpressing HeLa cells, reacidified lysosomal pH (10 min after NH_4_Cl washing) markedly decreased LC3 puncta, which is consistent with the fact that re-acidification decreased LC3-II levels in TPC2-overexpressing cells as shown in Fig. 7*F*. Interestingly, Rab7 failed to co-localize with the remaining LC3 puncta in these cells. We speculate that lysosomal reacidification in the majority of TPC2-overexpressing cells quickly relieves the fusion blockage of autophagosomes and lysosomes to form autolysosomes, thereby leading to the degradation of LC3-II and the quenching of GFP fluorescence. The remaining LC3 puncta in these cells likely represent the immature autophagosomes induced by the repetitive post NH_4_Cl washing. However, around ⅓ of TPC2-overexpressing cells still contained large numbers of LC3 puncta after removing NH_4_Cl from the medium, and Rab7 puncta were indeed co-localized with LC3-II in these cells (Fig. 8*D*). We reason that lysosomal reacidification in these cells might be slow and just start to recruit Rab7 to the autophagosomes but not yet induce the fusion of autophagosomes with lysosomes. Taken together, these results suggest that TPC2 signaling prevents the recruitment of Rab-7 to autophagosomes by alkalizing lysosomal pH to inhibit autophagosomal-lysosomal fusion.

**FIGURE 8.** **TPC2 prevents the recruitment of Rab-7 to autophagosomes in HeLa cells.** *A*, starvation (60 min) induced RFP-Rab7 puncta, which were colocalized with GFP-LC3 puncta (*left panel*) or Lamp1 puncta (*right panel*) in control HeLa cells. *B*, RFP-Rab7 puncta were colocalized with Lamp1 (*right panel*) but not with GFP-LC3 puncta in TPC2-overexpressing HeLa cells. *C*, removing NH_4_Cl (10 min) from medium decreased LC3 puncta in the majority (⅔) of TPC2-overexpressing cells pulsed with NH_4_Cl and RFP-Rab7 failed to colocalize to the remaining LC3 puncta. *D*, after washing out NH_4_Cl for 10 min, ⅓ of TPC2-overexpressing cells still contained large number of LC3 puncta, which were co-localized with RFP-Rab7. *Scale bar* = 10 μm.

The article "Two Pore Channel 2 (TPC2) Inhibits Autophagosomal-Lysosomal Fusion by Alkalinizing Lysosomal pH" was retracted in 2017. Reasons: fabricated or falsified images; manipulated images; ethical violations by an author.

##### TPC2 on General Endosomal-Lysosomal Degradation

Because the increase of lysosomal pH normally compromises the lysosomal activity, we assessed whether TPC2 signaling simply disrupts the general lysosomal functions to inhibit autophagy maturation. The processing of cathepsin L from the precursor form to its mature form has been commonly used as a marker for lysosomal activity, yet we found that the processing of cathepsin L was only slightly compromised in TPC2-overexpressing HeLa cells compared with that in control cells (Fig. 9*A*), which might be due to the fact that TPC2 overexpression just marginally increased lysosomal pH (Fig. 7*B*). Next, an epidermal growth factor receptor (EGFR) degradation assay was performed to examine whether the TPC2 signaling also affects the general endosomal-lysosomal pathway. In this assay both control and TPC2-overexpressing HeLa cells were treated with EGF. In principle, after EGF binds to its receptors (EGFR), the receptor complex undergoes endocytosis and is targeted to lysosomes where it is ultimately degraded. As shown in Fig. 9*B* and supplemental Fig. S6*A*, BAF inhibited EGF-triggered EGFR degradation in a dose-dependent manner, whereas TPC2 overexpression had little effect on it, which was similar to that in control cells. Finally, a DQ-BSA-green degradation assay was applied to measure the general endosomal-lysosomal degradation. DQ-BSA-green is a BSA labeled with a self-quenching fluorescent dye. After DQ-BSA-green is delivered to lysosomes via endocytosis, it is hydrolyzed into single dye-labeled peptides by lysosomal proteases, thereby relieving self-quenching, and the fluorescence can subsequently be monitored by flow cytometry. As shown in Fig. 9*C* and supplemental Fig. S6*B*, TPC2 overexpression also had little effect on BSA degradation, whereas BAF markedly inhibited it. Collectively, these results document that TPC2 signaling does not inhibit the general endosomal-lysosomal degradation.

**FIGURE 9.** **TPC2 did not inhibit general endosomal-lysosomal degradation in HeLa cells.** *A*, shown is processing of cathepsin L from the precursor form to its mature form in control or TPC2-overexpressing HeLa cells treated with or without bafilomycin for 1 or 3 h. *B*, TPC2 overexpression failed to change EGF-induced EGFR degradation, whereas BAF (100 nm) completely abolished it in HeLa cells. *C*, TPC2 overexpression did not inhibit the degradation of DQ-BSA-green in HeLa cells, whereas BAF (100 nm) markedly inhibited it.

The article "Two Pore Channel 2 (TPC2) Inhibits Autophagosomal-Lysosomal Fusion by Alkalinizing Lysosomal pH" was retracted in 2017. Reasons: fabricated or falsified images; manipulated images; ethical violations by an author.

## DISCUSSION

Here we provide definitive evidence that NAADP/TPC2 signaling induced the accumulation of matured autophagosomes by inhibiting autophagosomal-lysosomal fusion (Figs. 2–5). Perturbing TPC2/NAADP signaling by either TPC2 knockdown or the addition of an NAADP antagonist, on the other hand, facilitated the progression of autophagy by promoting the formation of autolysosomes (Figs. 3–5). Instead of affecting or functioning downstream of mTOR (Fig. 6, *A* and *B*), TPC2 signaling actually alkalinized lysosomal pH to suppress autophagosomal-lysosomal fusion (Fig. 7), likely by preventing the recruitment of Rab-7 to autophagosomes (Fig. 8). Yet TPC2 signaling had little effect on general endosomal-lysosomal degradation (Fig. 9).

The acidic milieu in lysosomes is generated by the V-ATPase, a multisubunit protein complex that pumps protons into the lysosomal lumen against an electrochemical gradient at the expense of ATP hydrolysis (70). The influx of protons into the lysosomal lumen also creates a lumen-positive membrane potential that, reciprocally, mitigates the ability of the V-ATPase to continue pumping protons. Thus, transporters for cation efflux or anion influx or both must be activated to maintain the balance of acidic pH and membrane potential inside lysosomes (71). Although Cl^−^ influx, possible via ClC-7 or CFTR (cystic fibrosis transmembrane conductance regulator), has been shown to dissipate the restrictive electrical gradient for lysosomal acidification (72, 73), whether Cl^−^ is the main counterion is debatable, and the identity of Cl^−^ transporters in lysosomes also remains controversial (71). Likewise, Ca^2+^, whose concentration in lysosomes is high and is partially dependent on H^+^ gradient (74), has been proposed to constitute another counterion pathway. TPC2, TRPM2, and TPML1 have all been shown to mediate Ca^2+^ release from lysosomes triggered by NAADP or ADPR (adenosine diphosphate ribose) (24, 36). Yet here we found that NAADP treatment or TPC2 overexpression increased lysosomal pH to inhibit autophagosomal-lysosomal fusion (Fig. 7), and chelating Ca^2+^ by BAPTA-AM (≥ 1 h treatment) relieved TPC2-induced accumulation of both LC3-II and p62 (Fig. 6, *C* and *D*), indicating that Ca^2+^ is required for NAADP/TPC2-induced lysosomal alkalinization and subsequent fusion blockage. These data further suggest that Ca^2+^ is not the counterion for maintaining high H^+^ in lysosomes, and the search for the real counterion pathway must continue.

The article "Two Pore Channel 2 (TPC2) Inhibits Autophagosomal-Lysosomal Fusion by Alkalinizing Lysosomal pH" was retracted in 2017. Reasons: fabricated or falsified images; manipulated images; ethical violations by an author.

Regarding how NAADP/TPC2-triggered Ca^2+^ release raises lysosomal pH, we speculate that either a putative Ca^2+^/H^+^ exchanger (75) or an unidentified lysosomal Ca^2+^ ATPase (76), similar to SERCA, or the coupling of several lysosomal proton-cation counter-transporters, such as sequential action of Ca^2+^/Na^+^ exchangers and Na^+^/H^+^ exchangers, can be activated to refill the lysosomal Ca^2+^ pools at the expense of proton efflux upon Ca^2+^ release from lysosomes via TPC2. Obviously, deciphering how Ca^2+^ enters lysosomes is the key to resolving this mystery. However, other than the V-ATPase, ion channels or transporters responsible for the formation of the unique ionic environment, *e.g.* Na^+^, Cl^−^, K^+^, and Ca^2+^, inside lysosomes remain unknown (75). A future lysosomal proteomics study should help in identifying the respective transporters.

Here we found that the HeLa cell line, an NAADP-incompetent line, can be reconstituted to be NAADP-competent by overexpressing a wild type, but not a pore-mutant, TPC2 (Fig. 1, *A* and *C*), and treatment of TPC2-overexpressing cells with Ned-19, a NAADP antagonist, markedly inhibited NAADP-induced Ca^2+^ release (Fig. 1*C*). Thus, these data provide unambiguous evidence that NAADP can activate TPC2 for Ca^2+^ release and echo the previous finding that TPC2 is an NAADP effector (26–31). Yet we also found that TPC2 overexpression in HeLa cells in the absence of exogenous NAADP treatment, already alkalinized lysosomal pH (Fig. 7, *A–D*) and inhibited autophagy maturation (Figs. 2–5). Although the effects of TPC2 overexpression might be due to endogenous NAADP, the effects of NAADP-AM on Ca^2+^ release (Fig. 1, *A* and *C*) and autophagy inhibition (Fig. 4*D* and supplemental Fig. S3*A*) in TPC2-overexpressing cells were transient. It has recently been shown that NAADP does not directly bind to TPC2, arguing that NAADP might first bind to accessory proteins within the TPC2 complex and subsequently activate TPC2 (40–42). Therefore, the effects of TPC2 overexpression in HeLa or mouse ES cells might be caused by accessory proteins in the TPC2 complex, and NAADP, induced by extracellular stimuli or cellular stress (25, 77), could bind to these accessory proteins to further activate TPC2. However, at this stage we still could not exclude the possibility that the effects of TPC2 overexpression are due to endogenous NAADP, as the transient effects of NAADP-AM might be due to its instability in aqueous solution (55).

Two recent papers found that TPC2 forms a Na^+^ channel in lysosomes that can be potentiated by phosphatidylinositol 3,5-disphosphate, an endolysosome-specific phosphoinositide, and inhibited by ATP (66, 78). It was proposed that high intracellular ATP levels enable mTOR to phosphorylate TPC2, thereby keeping it at a closed state. On the other hand, cell starvation results in lower ATP levels and dissociation of mTOR from TPC2, thus activating TPC2 to allow Na^+^ release from lysosomes (66). However, here we found that overexpression of a wild type, not a pore-mutant, TPC2 in cells maintained in nutrient-rich medium already alkalinized lysosomal pH and suppressed autophagosome-lysosome fusion (Figs. 2–5), suggesting that TPC2 in high ATP levels is already open. Starvation promoted autophagy, *e.g.* LC3-II induction and p62 degradation, in both control and TPC2-overexpressing cells (Figs. 3*A* and 6*A*), arguing that nutrient deprivation does not further activate TPC2 to inhibit autophagy progression. Thus these data suggested that TPC2 suppresses autophagosome-lysosome fusion independent of mTOR or ATP levels. However, the role of intracellular phosphatidylinositol 3,5-disphosphate or Na^+^ release from lysosome on TPC2-mediated autophagy inhibition remains to be determined.

The article "Two Pore Channel 2 (TPC2) Inhibits Autophagosomal-Lysosomal Fusion by Alkalinizing Lysosomal pH" was retracted in 2017. Reasons: fabricated or falsified images; manipulated images; ethical violations by an author.

Also notably, these two papers found that NAADP cannot activate TPC2 for Ca^2+^ release from lysosomes mainly by performing a patch clamp study on enlarged endolysosomes treated with vacuolin-1 (66, 78), which is contrary to some of results presented in this study and a body of work published previously (26–31). Further investigations are needed to resolve the controversy, and a recent study suggests that a GFP tagged on the N terminus of TPC1 disrupts NAADP action (79).

Interestingly, mutation of TPC2, M484L, or G734E has been associated with blond *versus* brown hair by genome-wide association studies for pigmentation (80). The melanosome, a lysosome-related organelle, is the site of synthesis and transport of melanin pigments, thereby providing tissues with color and photoprotection. In addition, autophagy and autophagy regulators have been shown to play roles in both the biogenesis of melanosomes and melanosome destruction (81). Therefore, it is of interest to assess whether and how the two identified TPC2 mutants affect melanosome biogenesis or destruction via autophagy related processes. Without doubt, TPC2 signaling could play roles in other autophagic-related cellular processes. Given that autophagy plays important roles in a wide variety of cellular processes and dysfunctional autophagy has been associated with many human diseases, it is important to further dissect the TPC2 signaling to identify novel regulators in this pathway. Development of novel reagents targeting TPC2 signaling, e.g. NAADP analogues, to manipulate autophagy should provide alternative pharmaceutical intervention in the treatment of autophagy-related human disorders. Along this line, Niemann-Pick disease, a human neurodegenerative lysosomal storage disorder, has been associated with abnormal lysosomal Ca^2+^ homeostasis, and its cellular phenotype is similar to that in TPC2-overexpressing cells (Fig. 2*A*) (29, 82). Whether TPC2-mediated autophagic regulation contributes to this disorder is, therefore, of great interest to pursue.

The article "Two Pore Channel 2 (TPC2) Inhibits Autophagosomal-Lysosomal Fusion by Alkalinizing Lysosomal pH" was retracted in 2017. Reasons: fabricated or falsified images; manipulated images; ethical violations by an author.

## Supplementary Material

Supplemental Data

## Footnotes

2 The abbreviations used are:

TPC2: two pore channel 2
NAADP: nicotinic acid adenine dinucleotide phosphate
tfLC3: RFP-GFP tandem-tagged LC3
BAF: bafilomycin-A1
EGFR: EGF receptor
ES: embryonic stem
WB: Western blot
RFP: red fluorescent protein
AM: acetoxymethyl
DQ: dye-quenched.
